# Assessment of the influence of whole body vibration on Cochlear function

This article has been retracted.

**DOI:** 10.1186/1745-6673-7-12

**Published:** 2012-06-21

**Authors:** Seyyed-Ali Moussavi-Najarkola, Ali Khavanin, Ramazan Mirzaei, Mojdeh Salehnia, Mehdi Akbari

**Affiliations:** 1 Department of Occupational Health, School of Medical Sciences, Tarbiat Modares University (TMU), Tehran, Iran; 2 Department of Occupational Health, Health promotion research center, Zahedan University of Medical Sciences (ZUMS), Zahedan, Iran; 3 Department of Anatomical Sciences, School of Medical Sciences, Tarbiat Modares University (TMU), Tehran, Iran; 4 Department of Audiology, School of Rehabilitation, Iran University of Medical Sciences (IUMS), Tehran, Iran

**Keywords:** Cochlear function, Whole body vibration, Distortion product otoacoustic emissions, Rabbit's hearing, DPOAEs

## Abstract

**Background:**

Whole body vibration (WBV) is a potentially harmful consequence resulting from the dissipation of energy by industrial machineries. The result of WBV exposure on the auditory system remains unknown. The objective of the present research was to evaluate the influence of WBV on cochlear function, in particular outer hair cell function. It is hypothesized that WBV impairs cochlear function resulting in decreased Distortion Product Otoacoustic Emission (DPOAE) levels (L_dp_) in rabbits subjected to WBV.

**Methods:**

Twelve rabbits were equally divided into vibration and control groups. Animals in vibration group were exposed to 1.0 ms^-2^ r.m.s vertical WBV at 4–8 Hz for 8 h/day during 5 consecutive days. Outer hair cell function was assessed by comparing repeated-measurements of DPOAE levels (L_dp_) across a range of f_2_ frequencies in rabbits both exposed and unexposed to WBV. DPOAE level shifts (LS_dp_) were compared across ears, frequencies, groups, and times.

**Results:**

No differences were seen over time in DPOAE levels in the non-exposed rabbits (p = 0.082). Post-exposure L_dp_ in rabbits exposed to WBV were significantly increased at all test frequencies in both ears compared to baseline measures (p = 0.021). The greatest increase in L_dp_ following exposure was seen at 5888.5 Hz (mean shift = 13.25 dB). Post-exposure L_dp_ in rabbits exposed to WBV were not significantly different between the right and left ears (p = 0.083).

**Conclusion:**

WBV impairs cochlear function resulting in increased DPOAE responses in rabbits exposed to WBV. DPOAE level shifts occurred over a wide range of frequencies following prolonged WBV in rabbits.

## Background

Many workers are unavoidably subjected to whole body vibration (WBV) due to the nature of assigned duties. WBV is frequently found in various industries and environments. Whole-body vibration (WBV) is caused by vibration transmitted through the seat or the feet by workplace machines and vehicles with frequencies of concern ranging from 0.5 to 80 Hz [1].

General health and well-being effects of WBV exposure on the human body have been studied over a number of years [2]. Both animal and human studies have shown that exposure to high levels of vibration can have serious effects on the human body, causing damage to a variety of vital organs [3]. WBV exposure may result in musculoskeletal impairments, central or peripheral nervous disorders [4]. Moreover, sympathic and gastrointestinal disorders are reported due to WBV [5].

Occupational deafness may be caused or aggravated by the additive effects of several environmental factors, especially vibration [6]. A paucity of studies has been conducted on the assessment of the influence of WBV exposure on cochlear function at non-realistic levels typically found in industrial settings. Okada *et al.* (1972) cited that temporary threshold shift (TTS) occurred after both 20 and 60 min of exposure to vibration with an acceleration of 500 cm/s and a frequency of 5 Hz, which is regarded as a resonance frequency of human body [7]. Yokoyama *et al.* (1974) showed that there was no significant change in threshold sensitivity after exposure to vibration alone [8]. While the literature on whole-body vibration is inconclusive, Hamernik *et al.* (1980) suggested that vibration may induce or increase hearing loss or cochlear damages. Based on their opinion, low frequencies (<100 Hz), although relatively ineffective in initiating an auditory response, can vibrate the membranous labyrinth if levels are high enough [9]. Hamernik *et al.* (1981) reported that vibration alone had essentially no effect on threshold [10]. While, Hamernik *et al.* (1989) showed that only stronger vibration exposure conditions (30-Hz, 3 g r.m.s) can alter the dependent measures of hearing and can alter the shape of the permanent threshold shift (PTS) audiogram [11]. Soliman *et al.* (2003) reported that the exposure to vibration only led to enhancement of both DPOAE amplitude and signal to noise ratio [12]. Bochnia *et al.* (2005) showed that vibration-induced damages to the inner ear structures may cause a worsening of hearing, especially at low and medium frequencies [13]. Therefore, a significant gap is evident in understanding the result of WBV exposure on cochlear function at realistic levels typically found in industrial settings.

Distortion Product Otoacoustic Emissions (DPOAEs) are sounds measured in the ear canal that reflect mechanical activity of outer hair cells [14]. In animals, DPOAEs can be used to screen hearing by providing an objective means of confirming healthy cochlear function [15]. DPOAEs are measured in response to two simultaneously presented primary tones, f_1_ and f_2_, where f_2_ is slightly higher in frequency and at a level equal to or less than f_1_[16]. DPOAEs are likely generated from at least two locations on the basilar membrane, the overlapping region between f_1_ and f_2_, nearer to the f_2_ place, and the cubic distortion place (2f_1_-f_2_) [17]. DPOAEs are most commonly measured as Distortion Product diagrams (DP-grams) that depict DPOAE levels (L_dp_) as a function of f_2_ for a selected combination of primary-tone levels L_1_ and L_2_[18,19].

The objective of the present study was to evaluate the influence of WBV on cochlear function, in particular outer hair cell function. It is hypothesized that WBV impairs cochlear function resulting in decreased DPOAE levels (L_dp_) in rabbits subjected to WBV.

## Materials and methods

### Laboratory animal model and animal house condition

Three months old, healthy male New Zealand White rabbits (weighing from 1800 to 2200 g; mean 2000 g) selected from Pasture Institute of Iran were divided into two groups as control (C) and vibration (WBV) groups. The sample size for the minimal effect size was calculated to be 5, while 10% should be added for probable death [20]. Thereby, total sample size was calculated at 5.5 and rounded to 6 (for each group). In the present study, 12 healthy rabbits were selected among 15 rabbits based on their hearing ability measured by DPOAE responses and were divided into two groups. Rabbits were maintained in a conditioned animal house at 20-22°C temperature, 30-70% relative humidity, and 10 times/h air exchange. Animals were kept on a 12-h light/12-h dark cycle. Required space for each rabbit by 2000 g body weight was considered about 0.14 m^2^ according to toxicology reference conditions [20]. Rabbits were allowed free access to food (Pars laboratory animal chow) and tap water. "General Principles of Helsinki Law related to Laboratory Animal" were followed.

### Exposure protocol

Experimental animals were subjected to 1.0 ms^-2^ r.m.s (root mean square) WBV in z-axis at 4–8 Hz for 8 h per day during 5 consecutive days by putting them into an exposure chamber on a vibrating platform, while control animals were treated identically except exposure to WBV. Experimental protocol was set as: pre- DP-gram (baseline; day 0), rest periods (3 days on days 1 to 3), exposure periods (only for vibration rabbits; WBV exposure on days 4 to 8), first post- DP-gram (immediately following WBV exposure); rest period (3 days; days 9 through 11), and second post- DP-gram (72 h following WBV exposure).

### WBV exposure chamber

Six experimental rabbits were exposed to vertical WBV with definite characteristics by putting them into a 50 × 50 × 50 cm transparent poly carbonate Plexiglas chamber on a self constructed vibrating platform (Figure 1). Vertical vibration (in z-axis) was chosen to achieve a larger pathway, longer stability and more impact for passing WBV along the body and implemented according to ISO-2631 (1997). Like other general vibrating systems, this system also consisted of three components including mass (total mass of chamber, 8 spring shock absorbers, metal plate dimensioned 50 × 50 cm, mounts, rabbits' weights, and 4 compressed plastic shock absorbers was equal to around 45 kg), stiffness (spring and shock absorbers), and damping. Vibrating platform was formed from a three-phase body vibrator (Model M3/65, ITAL VIBREH Company; Italy) for generating vibration and an inverter (Model 0.37 KW IG5A-4; LG Company; Korea) to obtain to desired characteristics of WBV. Air displacement was about 10 times/h by allocating 20 openings with a 3 cm diameter at the lateral faces and floor as well as 2 windows dimensioned 10 × 15 cm at the ceiling. Laboratory background noise was monitored systematically during experiments with a Casella CEL-490 sound level meter located near the exposure chamber. Background noise in the animal house and lab was found to be below 20±2 dBA SPL.

**Figure 1:** **Plexiglas exposure chamber inserted on a vibrating platform.** The vibrating system consisted of mass, stiffness (spring and shock absorbers), and damping, with a total mass of 45 kilograms.

### DPOAE examinations

At the end of the exposure period, rabbits were anaesthetized by intramuscular injection of 60% Ketamine (40 mg/kg, i.m.) and 40% Xylazine (10 mg/kg, i.m.) mixture. Before DPOAE measurement, animals were examined otologically to exclude any infection and/or remove ear channel blocking wax. At the time of DPOAE recordings, middle ear function was examined by tympanometry test (226-Hz tympanometry, with an 85 dB sound pressure level: SPL, and 400 daPa/s; Madsen-Zodiac 901; GN Otometrics, Münster Company, Germany). The criteria for normal middle-ear function were set as Type-A tympanogram, middle ear pressure values between −100 and +50 daPa, and middle ear compliance values between 0.3 and 2.0 ml. DPOAE analyzer (DPOAE 4000 I/O Model; made of HOMOTH Company; Germany) were used for recording the outer hair cells function in both ears of the animals. DPOAEs were measured in an acoustic room with background noise level less than 3 dBA SPL. Two pure primary tones (L_1_ = 75 and L_2_ = 65 dB SPL; L_1_-L_2_ = 10 dB SPL) with f_2_/f_1_ = 1.25 were used to measure DPOAEs at f_2_ frequencies ranging from 500 Hz to 10 kHz. Ten f_2_ frequencies were measured as the best auditory sensitivity responses in NZW rabbits due to classical conditioning of the nictitating membrane (NM) response [21]. The criterion for normal DPOAE was defined so that the difference between the emission level and the noise-floor levels (SNR) was above 6 dB SPL. Before DPOAEs, signal levels were calibrated in the ear canal by an emission probe microphone. The contents of stimuli were summed, and the summed energy in the 2f_1_–f_2_ frequency buffer was served to estimate DPOAE amplitudes. DPOAE levels (L_dp_) on three occasions were examined, and their respective level shifts (LS_dp_) were compared between control and WBV groups. Constant body temperature was controlled during the DPOAE examinations for avoiding intervention in measurements.

### Statistical analysis

Two-sample Kolmogorov-Smirnov analysis was used to assess the normality of collected data. Power analysis was used to calculate the minimum sample size required to get a significant result (H_0_:$\bar{x}$=6). Repeated measures analysis of variance (ANOVA) was used to compare L_dp_ across test sessions within each group. One-way ANOVA was used to compare L_dp_ between groups at each test session, and post-hoc comparisons were adjusted when necessary using Tukey’s Honestly Significant Difference. Paired-sample T-test was used to compare L_dp_ between the right and left ears. Independent-Sample T-test was used to compare L_dp_ across pre- and post-exposure times. Differences were considered significant with p < 0.05.

## Results

Collected data was confirmed to be normal in both the control and WBV groups (C.I. = 0.95; Z = 328; p < 0.001). The sample size of the study design was adequate to achieve significance at an effect size of 83.6% of the normal signal.

Pre- and post-exposure DPOAE analyses revealed that no differences were seen over time in DPOAE levels (L_dp_) in the non-exposed rabbits (F = 4.72; p = 0.082) (Figure 2a,b). L_dp_ were not significantly different between the right and left ears (t = 3.13; p = 0.076), nor were they different across frequencies (F = 6.21; p = 0.063).

**Figure 2:** **DPOAE levels and noise floor levels in control rabbits.** L_dp_ and L_nf_ were measured in control and WBV exposed rabbits, with L_1_ = 75 dBA, L_2_ = 65 dBA and a f_2_/f_1_ ratio of 1.25. **a:** right ear; **b:** left ear. Each point represents mean±1 SD from 6 rabbits.

DPOAE level (L_dp_) analyses showed that the pre-exposed L_dp_ of rabbits in WBV group were found to be equal to those measured in control rabbits (p = 0.089) (Figure 3a,b), while post-exposure L_dp_ in rabbits exposed to WBV were significantly increased at all test frequencies in both ears as compared to the respective controls (t = 3.48; p = 0.035) or in rabbits prior to exposure (t = 5.25; p = 0.021). The greatest post-exposure L_dp_ was seen at 5888.5 Hz (mean L_dp_, _day 8_ = 49.72 dB; mean L_dp_, _day 11_ = 46.19 dB). Post-exposure L_dp_ in rabbits exposed to WBV were not shown to be significantly different between the right and left ears (t = 5.78; p = 0.083).

**Figure 3:** **DPOAEs levels and noise floor levels in WBV exposed rabbits.** Experimental conditions are identical to those described in Figure 2.

First and second DPOAE level shifts (LS_dp_) in WBV rabbits were found to be significantly different from those measured in the respective controls (p = 0.019 and p = 0.023 respectively) (Figure 4a,b). LS_dp_ following exposure to WBV were significantly different across times (F = 4.77; p = 0.031). The greatest first and second LS_dp_ (the greatest increases in L_dp_, _day 8_ and L_dp_, _day 11_) in rabbits following exposed to WBV were shown at 5888.5 Hz (mean first level shift = 13.25 dB, mean second level shift = 10.8 dB). LS_dp_ in rabbits subjected to WBV were not significantly different between the right and left ears (p = 0.075).

**Figure 4:** **First and second DPOAE**_**s**_**level shifts (LS**_**dp**_**) in control and WBV exposed rabbits.a**: right ear; **b**: left ear.

## Discussion

DPOAE levels (L_dp_) in vibration rabbits were increased at a vast range of frequencies, mostly at mid-to-high frequencies (i.e., L_dp_ increased slowly from 588 Hz to 5888.50 Hz, then decreased steeply to 9855 Hz). There are, therefore, two important findings in this study: 1) WBV resulted in DPOAE level (L_dp_) increases, and; 2) the greatest change in DPOAE level (L_dp_) occurred at 5888.5 Hz. Consistently, Soliman *et al.* (2003) showed that 4-weeks-exposure to vibration only in guinea pigs led to enhancement of DPOAE amplitudes [12]. Martin *et al.* (1977) reported that NZW rabbits’ auditory sensitivity is maximal in the mid-to-high frequency range and rapidly decreased in the lower and higher frequencies due to the conditional nictitating membrane (NM) response [21]. Deviating from our finding, Soliman *et al.* (2003) found the maximum DPOAE response amplitudes in WBV guinea pigs at 1006 Hz [12]. Brown (1987) believed that DPOAE levels (L_dp_) tend to be largest at the frequency of the highest hearing sensitivity in the animal species [22]. Soliman *et al.* (2003) concluded that more damage to the inner hair cells than the outer hair cells is the reason for increased DPOAE amplitudes in WBV exposed animals [12]. These increments were believed to be related to the affected IHC_s_ by loss of afferent input which reduced the activity in the efferent olivocochlear bundle as well as the presence of normal OHC_s_ that amplified the generation of DPOAEs [12]. Similar studies proposed different effects of WBV exposure on the cochlear function through a variety of causes. Okada *et al.* (1972) reported temporary threshold shift (TTS) after vibration exposure, which were suggested to occur at the resonance frequency of human body [7]. Temkin (1973) showed that vibration is responsible for increasing cochlear damage from noise exposure in mice [10]. Hamernik *et al.* (1989) found that histological changes in the extent of the outer hair cell loss were responsible for the cochlear function shifts that occurred following vibration exposure conditions [11]. Bochnia *et al.* (2005) asserted that vibration-induced changes were seen in all the examined inner ear areas, whereas hair-cell damage was more often seen in the apex, spreading gradually to the base and from the circumference (outer hair cells of the third row) to the modiolus [13]. Hamernik *et al.* (1980) found that a damaged cochlea and vibrated membranous labyrinth were the main causes for vibration-induced cochlear function changes after low-frequency vibration [9]. Consistent with the results of this study, several factors were found to be associated with the enhanced DPOAE response amplitudes such as hypoxia [23], low frequency electromagnetic fields [24,25], and induced labyrinthitis [26,27], and some ototoxic drugs [26]. By contrast, some other studies reported that the DPOAE response amplitudes were significantly depressed following a number of factors including the administration of ototoxic drugs [28,29], acoustic trauma or noise overexposure [29,30], Meniere’s disease [31], sudden idiopathic sensorineural hearing loss [32], acoustic neuroma [33], presbycusis [34], and hereditary hearing disorders [35].

DPOAE levels (L_dp_) were found to change with the time after exposure. L_dp_ was elevated on day 8, then decreased to a level slightly higher than baseline on day 11. Similar reversible and temporary differences were reported after interrupting the exposure to different noxious agents such as noise overexposure or acoustic trauma [30], ototoxic drugs [28], sudden idiopathic sensorineural hearing loss [32], and thermoprobe lesioning [36]. These increases in DPOAE levels (L_dp_) might be attributed to the temporary and reversible effect of the vibration exposure as a basal cochlear lesion progressed through the frequency region being monitored. Consistently, other data confirm that the temporary increase in DPOAE amplitudes occurring before reductions can be interpreted as an improvement of the general condition of the exposed rabbits over time [26,37]. This could be interpreted that with continued DPOAE monitoring, the emissions would eventually return to baseline values as indicted by the decrease in the LS_dp_ between days 8 and 11. This also may be related to the presence of a lesion more basal than the frequency region being monitored [26] and the reversible recovery from temporary OHC_s_ fatigue [12]. This released OHCs from the suppression leads to DPOAE amplification, so that DPOAE somewhat returns to the normal values after recovery from vibration, coinciding with disappearance of vacuolation from IHCs. This will results in the return of olivocochlear bundle activity, with normalization of OHC activity [12].

DPOAE levels (L_dp_) in vibration-exposed rabbits were not found to be significantly different across the ears. The same vibration exposure, as well as the presence of a little distance between the rabbit's seat and the vibration generator seemed to be the main reason for the identical findings on two ears. Consistent with this result, some studies confirmed that DPOAE amplitudes were the same on right and left ears [2,3,12]. Contrary to this finding, pitch discrepancy (binaural diplacusis) were reported across the ears while presenting the same frequency stimulus [38], and tone-evoked DPOAE amplitudes were somewhat larger in the left ear [39]. Efferent activity seemed to be involved in the systematic binaural discrepancies of DPOAE response magnitudes on right and left ears in humans [40].

First and second DPOAE level shifts (LS_dp_) in rabbits subjected to vibration were found to be distinctly larger than those measured in rabbits not exposed to vibration. Similar finding appeared in guinea pigs at LS_dp_ following a 4-week vibration exposure that could be attributed to the normal OHC_s_, severely vacuolated IHC_s_, and edematous and vacuolated supporting cells [12].

## Conclusion

WBV impairs cochlear function resulting in increased DPOAE responses in rabbits. DPOAE level shifts occurred over a wide range of frequencies following prolonged WBV. WBV caused first DPOAE level shifts on day 8 which transformed to second DPOAE level shifts on day 11 because of partial reversible recovery following interruption of exposure. Increased understanding of the physiology of enhanced DPOAE levels (L_dp_) in rabbits will require a parallel histological study.

## Competing interests

The authors declare that they have no competing interests.

## Authors' contributions

SAMN, AK, RM and MS contributed to the conception, design and drafting of this manuscript. SAMN also carried out the audiometry tests, participated in the sequence alignment of the drafted manuscript, performed experiments and analyzed audiometry data. MA performed the calibration and setting of the DPOAEs device prior to audiometry test. All authors read and approved the final manuscript.
